The article "Skin Cancer Detection Using Kernel Fuzzy C-Means and Improved Neural Network Optimization Algorithm" was published in 2021. Journal: Comput Intell Neurosci.

# Skin Cancer Detection Using Kernel Fuzzy C-Means and Improved Neural Network Optimization Algorithm

**DOI:** 10.1155/2021/9651957

**Published:** 2021-07-17

**Authors:** Jia Huaping, Zhao Junlong, A. M. Norouzzadeh Gil Molk

**Affiliations:** ^1^College of Computer, Weinan Normal University, Weinan, Shaanxi, China; ^2^Rehabilitation Medicine Department, Weinan Central Hospital, Weinan, Shaanxi, China; ^3^Department of Computer Engineering, University of Guilan, Rasht, Iran

## Abstract

Early diagnosis of malignant skin cancer from images is a significant part of the cancer treatment process. One of the principal purposes of this research is to propose a pipeline methodology for an optimum computer-aided diagnosis of skin cancers. The method contains four main stages. The first stage is to perform a preprocessing based on noise reduction and contrast enhancement. The second stage is to segment the region of interest (ROI). This study uses kernel fuzzy C-means for ROI segmentation. Then, some features from the ROI are extracted, and then, a feature selection is used for selecting the best ones. The selected features are then injected into a support vector machine (SVM) for final identification. One important part of the contribution in this study is to propose a developed version of a new metaheuristic, named neural network optimization algorithm, to optimize both parts of feature selection and SVM classifier. Comparison results of the method with 5 state-of-the-art methods showed the approach's higher superiority toward the others.

## 1. Introduction

Cancer is fundamentally an uncontrolled cell division disease. Its growth is usually associated with a group of variations in the action of the cell cycle regularized. The inhibitors of the cell cycle stop cell division while situations are not proper; therefore, so little action of these inhibitors can cause cancer. Cancer cells disregard the signals that must cause cells to prevent dividing. For example, when common cells growing in a culture medium are surrounded on all sides by adjacent cells, they no longer divide (contact inhibition). On the contrary, cancer cells divide into layers in a mass and stack on top of each other, and contact inhibition does not prevent them from growing. One of the most dangerous cancers around the world is skin cancer. The skin, as the first cell layer of the body that is in connection with the outside environment, can suffer from many injuries and diseases. The most common cancer in the United States is skin cancer, which happens in the tissues of the largest section of the skin body. Skin cancer generally occurs on the outer layer of the skin, which may first appear as a swelling, bulge, or different section of the skin [1]. The skin blocks heat, sunlight, sores, and infections; it also warms the body and stores fat water in the body and produces vitamin D. The skin owns 2 principal layers: the superficial layer of the skin (epidermis) and the inner skin (dermis) [2]. The skin's surface layer (epidermis) is mainly composed of flat, scaly cells named Squamous cells. Round cells, called basal cells, are located beneath the superficial cells of the squamous melanocyte in the surface layer [3]. Prolonged exposure to sunlight enhances melanoma skin cancer's risk over a lifetime. One of the most dangerous kinds of cancer is Melanoma, which is caused by damage caused by overexposure to the sun and some other factors. Melanoma can be diagnosed with skin biopsies.  Figure 1 shows the statistical information of the lead cancers in quantity and death value in 2019 [4].

The article "Skin Cancer Detection Using Kernel Fuzzy C-Means and Improved Neural Network Optimization Algorithm" was published in 2021. Journal: Comput Intell Neurosci.

If melanoma is diagnosed and treated early, it can be treated, and late diagnosis can lead to the patient's death. Only experienced physicians can diagnose melanoma on time using appropriate tools and histological reports. One of the devices used to diagnose melanoma is dermatoscopy. With this tool, changes in the pigmentation of skin lesions in diseases can be evaluated. With the development of science in recent years, digital dermatoscopy has been replaced by conventional dermatoscopes with the ability to capture and store skin images. With the development of digital dermatoscopes, the development of an algorithm for the diagnosis of melanoma was considered by researchers, and then, other methods were proposed to enhance the accuracy of skin lesion diagnosis. Some of the selected researches are explained in the following.

Astorino et al. [5] suggested an approach for melanoma diagnosis. The method uses multiple instance learning (MIL) approach on some dermoscopy images to categorize between melanomas and common nevi. The method was then analyzed by comparing it with some state-of-the-art classification methods, like support vector machine. Simulation outcomes demonstrated that the suggested approach accomplishes better precision. A leave-one-out authentication is carried out on a dataset and showed the method's higher efficiency.

Mohamed et al. [6] suggested an image processing approach for melanoma diagnosis. The method used a simple pipeline image preprocessing technique including methods like image conversion, noise reduction, and hair removal. Also, the melanoma area is threshold to segment the area, and then, feature extraction was used for taking out the main features of the image using the ABCD rule.

Barros et al. [7] proposed a real-time cancer diagnosis system based on hardware designing by the field-programmable gate arrays (FPGA). A multilayer perceptron artificial neural networks (ANN) is utilized for this purpose. The proposed image processing is used to extract the characteristics of the skin from the images and classify them based on the features and using the ANN classifier. Simulation results of the proposed approach are confirmed by an open-access database. Ultimate results of the suggested approach were then compared with the results of another hardware-based technique using ARM A9 microprocessor to demonstrate the method's proper performance.

The article "Skin Cancer Detection Using Kernel Fuzzy C-Means and Improved Neural Network Optimization Algorithm" was published in 2021. Journal: Comput Intell Neurosci.

Santos and Espitia [8] presented an approach for the diagnosis of uveal melanoma (UM), which is a sort of intraocular cancer. The suggested technique combined iris segmentation methods and designed a method for UM diagnosis based on neural networks and fuzzy logic. Simulation results of the study indicated 96.04% accuracy for the artificial neural networks and 76% correct classification for the fuzzy logic system.

Wang [9] proposed an all-inclusive method to provide a proper segmentation technique. The method is applied based on deep convolution networks on the hyperspectral pathology images. The study employed a 3D fully convolutional network, called Hyper-net, to obtain the best performances of segmentation from the hyperspectral pathology images. The loss function was then modified for improving the model sensitivity. Ultimate outcomes demonstrated that the suggested approach has higher performance than the 2D models in the aim of segmentation.

The present research suggests a novel optimized pipeline methodology for automatic detection of skin cancer detection. The method includes four main phases. The first phase is preprocessing of the input image to prepare it for the main processing. The first phase here includes two parts: noise reduction and contrast enhancement. The next phase is to segment the region of interest. Afterwards, the features are extracted, and the best ones selected for injecting to a support vector machine (SVM) as the final phase. This investigation employs an improved version of a new metaheuristic, called neural network optimization algorithm, to optimize both parts of feature selection and SVM classifier. This can improve the accuracy of the system as can be seen in the next sections. The main contribution of the paper has been highlighted as follows:

- An early diagnosis system for skin cancer from dermoscopy images is proposed
- Kernel fuzzy C-means is used to segment the region of interest (ROI)
- Some features from the ROI are extracted for the final diagnosis
- An improved neural network algorithm is used for optimal feature selection
- Support vector machine (SVM) is used for final classification
- Comparison results are compared with 5 state-of-the-art methods

Figure 2 illustrates the flowchart of the suggested approach.

The article "Skin Cancer Detection Using Kernel Fuzzy C-Means and Improved Neural Network Optimization Algorithm" was published in 2021. Journal: Comput Intell Neurosci.

## 2. Image Preprocessing

### 2.1. Noise Reduction

Ordinary nonpolarized light is used in medical images. Since, according to “Fresnel relations,” the reflection of light from the surface of matter and its underlying layers and scattering from uneven and rough surfaces is affected, as well as a function of the state of polarization of light, it is possible to eliminate some annoying and destructive reflected or diffused lights by using a suitable filter to achieve a high signal to noise ratio. Therefore, the first step for starting the image analysis of the cancer images is to eliminate, or, at least, reduce, this noise to have a high quality of images for processing. Different methods have been introduced for this purpose. One simple and popular method for noise reduction is Median filtering. However, this filter is nonlinear; it has some significant advantages such as

keeping the main edges of the image after filtering. In the median filter, the pixels have been substituted by the median value of their neighbors, i.e.,

(1) $$\begin{array}{c} Z_{m,n}=\text{median }\left(y_{i,j}:\left(i,j\right)\in \beta \right), \end{array}$$

where *β* signifies the neighborhood of the considered pixel in position (*m*, *n*).

The present study uses a 3 × 3 mask for the median filter. This selection is based on trial and error and may be different for other databases. Thus, it should be the point that using a higher mask can improve the probability of edges losing.  Figure 3 shows an example of using the median filtering for noise reduction of the input images with considering 0.1 noise density salt and pepper noises.

### 2.2. Contrast Enhancement

In some situations, due to different reasons, like the sufficient user experience's lack in imaging and the bad quality of measurement devices and sensors utilized in them, the contrast of the images has lessened, such that its intensity gets darkened, or overexposed. To correct this deficiency from the images, we need to implement the image contrast enhancement. Therefore, in this study, we can use an image contrast enhancement step on the low-quality images to improve the image contrast to simplify the segmentation step. The present study considers global contrast enhancement based on Lookup Table to reach this purpose [10]. The method of global contrast enhancement is formulated as follows:

(2) $$\begin{array}{c} {\text{Out}}_{H}=\frac{{\text{In}}_{H}-{\text{Min}}_{H}}{{\text{Max}}_{H}-{\text{Min}}_{H}}, \end{array}$$

where Out_*H*_ signifies the improved output image, and Min_*H*_ and Max_*H*_ demonstrate the minimum and the maximum levels of gray values of the original image histogram, orderly. We used an 8-bit lookup table for the method. A simple contrast enhancement on a medical image is shown in Figure 4.

The article "Skin Cancer Detection Using Kernel Fuzzy C-Means and Improved Neural Network Optimization Algorithm" was published in 2021. Journal: Comput Intell Neurosci.

## 3. Medical Image Processing

### 3.1. Segmentation Based on Kernel-Based Fuzzy C-Means

One of the significant issues in medical image processing is the image segmentation of the medical image into its components. Image segmentation describes the success or the final failure of image analysis methods. However, there is no general method for successful segmentation of all medical images, and it still has good research areas due to its wide application. The accuracy of this study is crucial in areas such as medicine, which helps preserve and protect human life. Due to the wide range of applications, it provides image segmentation and the use of methods in various fields.

The importance of this part especially in mammographic images is too high, because medical images have a naturally low quality, which makes them a complicated problem for mass segmentation. This research uses an enhanced multistep fuzzy C-means method for performing on the skin cancer images for their mass segmentation. Based on this method, the first step is to generate superpixels using a simple linear iterative clustering (SLIC) algorithm [11]. The SLIC algorithm generates superpixels based on CIE LAB color space in 5D space. Afterwards, texture and color properties are employed to separate the superpixels and finally to find the image elements.

Then, the color feature from the superpixels has been extracted and has been arranged, such that, for all images in HSV space, three separate histograms for S, H, and V channels have been considered. To reduce time complexity, the histograms have been quantized into 8, 4, and 2 subdistances. Afterward, to find the texture features, the NSCT algorithm has been used. Then, the generated data is clustered by a fuzzy kernel, and all superpixels with cluster tags have been placed in one cluster. This study uses kernel fuzzy C-means (KFCM) algorithm employing segmentation. This technique offers a kernel-based version of fuzzy C-means to evaluate the data point's distance from the center of clusters. The kernel function in this study is achieved as follows:

(3) $$\begin{array}{c} K=\exp\left(\frac{-x-y^{2}}{\rho }\right). \end{array}$$

First, the membership function has been evaluated. Then, based on a similarity measure of kernel fuzzy, the belonging of each data sample to the clusters has been achieved. The pseudocode of the algorithm is given as follows:

(1) Apply KFCM to cluster the set of objects and generating a *U* membership matrix [12]
(2) In all elements, *x*_*i*_, *x*_*j*_, the number of *t* nearest neighbor is found.
(3) If *x*_*i*_, *x*_*j*_ are not *t* nearest neighborhood, *W*_*ij*_=0.
(4) Else if they belong to a cluster, *W*_*ij*_=1.
(5) Else, *W*_*ij*_=exp(*ln*2 × (*u*_*i*_ ⊕ *u*_*j*_)), where ⊕ defines the exclusive OR that totally indicates the overlap between two fuzzy sets.
(6) Here, diagonal matrix, *D*, is formulated as follows:
  (4) $$\begin{array}{c} D_{ij}=\sum_{j=1}^{n}W_{ij}. \end{array}$$
And, it is normalized as follows:
  (5) $$\begin{array}{c} L=D^{-1/2}{\text{WD}}^{1/2}. \end{array}$$
The number of *K* bigger eigenvector than *L* (the first vector) is found (the first vector is selected), and the matrix *P*=[*p*^1^, *p*^2^,…, *p*^*k*^] has been formed, and then, the algorithm normalizes the rows in the *P* matrix to form matrix *Y*.
(7) Each line of *Y* has considered a point in space *R*^*k*^ and at then, the final clustering has been established by the K-means algorithm.

Figure 5 shows two sample examples of skin cancer segmentation based on the proposed KFCM methodology.

The article "Skin Cancer Detection Using Kernel Fuzzy C-Means and Improved Neural Network Optimization Algorithm" was published in 2021. Journal: Comput Intell Neurosci.

## 4. Improved Neural Network Algorithm

### 4.1. Optimization

Generally speaking, in most applications of engineering, optimization is a vital subject. Optimization is to make the best decision to get the optimal (minimum or maximum) result for the considered problem. Several methods have been introduced for optimization. However, classic methods as exact methods can solve these problems, and they fail in some cases that the problem is nonlinear or complicated. To overcome this problem, another technique, called metaheuristic, has been introduced [13]. Metaheuristics include a set of optimization algorithms that are inspired by nature, human behaviors, animals' competitions, etc. The main advantage of using metaheuristic algorithms is that they use random structure instead of using gradient methods. This simplifies the optimization process [14]. Furthermore, the most complicated problems are that their number is increasing day by day and they cannot be solved by the classic methods, but these methods, based on their stochastic nature, can find a near-optimal result in a logical time. There are different types of these algorithms like ant lion optimizer (ALO) algorithm [15], chimp optimization (CO) algorithm [16], Harris Hawks optimization [17], and world cup optimization (WCO) algorithm [18]. Recently, a new metaheuristic algorithm, called neural network algorithm (NNA), is introduced, which is inspired by the concepts of biological nervous systems and artificial neural networks (ANNs). Based on [19], each ANN includes some artificial neurons, which are inspired by the biological nervous systems. The relationships among units principally specify the network function. The NNA approach is illustrated in the following.

The article "Skin Cancer Detection Using Kernel Fuzzy C-Means and Improved Neural Network Optimization Algorithm" was published in 2021. Journal: Comput Intell Neurosci.

### 4.2. Neural Network Algorithm

Like any other metaheuristic algorithm, the NNA starts with an initial population that is called the pattern. In NNA, just like ANN, the main idea is to update the pattern population to minimize error among the forecasted data and the desired output data. Here, the best solution is the desired output that can be updated in each iteration for achieving the minimum error amount by moving the pattern population in the direction of the desired solution. In the following, the algorithm methodology is briefly explained.

#### 4.2.1. Initialization

The first operation in this algorithm, like any other metaheuristic, is to generate some random population (decision variables) for initial evaluation. By considering a D dimensional problem, the considered pattern solution vector will be an array of 1 × D, representing input data in the NNA. Moreover, by considering the D dimension and *N*_pop_ several random candidates, the initial pattern population can be considered as follows:

(6) $$\begin{array}{c} X=\left[\begin{array}{cccc} x_{1}^{1} & x_{2}^{1} & \ldots & x_{D}^{1}\\ x_{1}^{2} & x_{2}^{2} & x_{3}^{2} & x_{D}^{2}\\ \vdots & \vdots & \ddots & \vdots \\ x_{D}^{N_{\text{pop}}} & x_{D}^{N_{\text{pop}}} & \ldots & x_{D}^{N_{\text{pop}}} \end{array}\right], \end{array}$$

where the matrix *X* is made randomly between the minimum and maximum limitations of a problem.

And, the cost value is achieved as follows:

(7) $$\begin{array}{c} C_{i}=f\left(x_{1}^{i},x_{2}^{i},\ldots ,x_{D}^{i}\right), \end{array}$$

where *f* describes the objective value.

After evaluating the objective value of each pattern solution, the best one is selected as the best pattern solution. The NNA has *N*_pop_ input data and *D* dimension with only one target data.  Figure 6 shows this structure.

After defining the target solution (*X*^*T*^) among the other pattern solutions, its weight (*W*^*T*^) has to be chosen from the population of weight (weight matrix).

In an ANN, the neurons connect with dendrite using a simple summation. The output is connected to the input layers based on weighted (*w*) interconnection. Initial weights are random values in this algorithm, and then, they have been updated based on some equations to provide the minimum network error. The initial weights in the algorithm are as follows:

(8) $$\begin{array}{c} W\left(t\right)={\left[\begin{array}{ccccc} w_{11} & \ldots & w_{i1} & \ldots & w_{N_{\text{pop}}1}\\ w_{12} & \ldots & w_{i2} & \ldots & w_{N_{\text{pop}}2}\\ \vdots & \vdots & \vdots & \vdots & \vdots \\ w_{1N_{\text{pop}}} & \cdots & w_{iN_{\text{pop}}} & \ldots & w_{N_{\text{pop}}N_{\text{pop}}} \end{array}\right]}_{N_{\text{pop}}\times N_{\text{pop}}}, \end{array}$$

where *W* includes uniformly distributer random values in the range [0, 1]. The first and the second subscripts of weight relate to the pattern solution and participated with the other solutions of the pattern. All pattern solutions have their weight value to generate a new candidate solution. These weights have also a constraint that should not exceed 1 and mathematically formulated as follows:

(9) $$\begin{array}{c} \sum_{j=1}^{N_{\text{pop}}}w_{ij}\left(t\right)=1,\;\\ w_{ij}\in U\left(0,1\right), \end{array}$$

where *i*, *j*=1,2,…, *N*_pop_.

The article "Skin Cancer Detection Using Kernel Fuzzy C-Means and Improved Neural Network Optimization Algorithm" was published in 2021. Journal: Comput Intell Neurosci.

Weight is randomly distributed values in the range between 0 and 1, where their aggregate in a solution of the pattern must not be more than one, which is because of the bias control of the movement and to generate the new pattern solutions. If the constraint is not considered, the probability of sticking in the local optimum by the values of the weight will be increased. After weight matrix formation, new pattern solutions (*X*^*N*^) are evaluated as follows:

(10) $$\begin{array}{c} X_{j}^{\text{New}}\left(t+1\right)=\sum_{i=1}^{N_{\text{pop}}}w_{ij}\left(t\right)\times X_{i}\left(t\right),\\ X_{i}\left(t+1\right)=X_{i}\left(t\right)+X_{i}^{\text{New}}\left(t+1\right). \end{array}$$

After achieving the new pattern solutions using the best weight amount that is named target weight, this updating is established by the following equation:

(11) $$\begin{array}{c} W_{i}^{\text{updated}}\left(t+1\right)=W_{i}\left(t\right)+2\times \text{rand}\times \left(W^{\text{Target}}\left(t\right)-W_{I}\left(t\right)\right). \end{array}$$

Another operator for updating in NNA is the bias operator. This operator is employed for modifying the exploration part of the algorithm by using a specific percentage of the candidates in the new population (*X*_*i*_^New^(*t*+1)) and updated weight matrix (*W*_*i*_^updated^(*t*+1)). The pseudocode of this operator is as follows:

  For I = 1 to *N*_pop_
  If rand ≤ *γ*
 
*N*_b_ = round (*D* × *γ*)
  For *j* = 1: *N*_b_
  X_Input_(I, integer rand [0, D]) = LB + (UB−LB) × rand.
  End for
 
*N*_wb_ = round (*N*_pop_ × *γ*)
  For *j* = 1: *N*_wb_
 
*W*^Updated^(*j*, integer rand [0, *N*_pop_]) = U (0,1).
  End for
  End if
  End for

Here, LB and UB represent the problem minimum and maximum bounds, orderly. *γ* describes the modification factor that defines the candidates' percentage. *γ*=1 at first, and then, it decreases gradually during the process based on any decreasing formulation as follows:

(12) $$\begin{array}{c} \gamma \left(t+1\right)=0.99\times \gamma \left(t\right). \end{array}$$

In the NNA, there is also a transfer function operator to transfer the new candidates to the new updated positions to provide better value against the target solution. The solution reimproved by giving the novel pattern solutions to the best solution direction (target solution). The transfer function operator (TF) can be formulated as follows:

(13) $$\begin{array}{c} X_{i}^{*}\left(t+1\right)=\text{TF}\left(X_{i}\left(t+1\right)\right)=X_{i}\left(t+1\right)+2\times \text{rand}\times \left(X^{\text{Target}}\left(t\right)-W_{i}\left(t+1\right)\right). \end{array}$$

The pseudocode of the collaboration between bias and TF operators is tabulated below:

  For *i* = 1 to *N*_pop_
  If rand ≤ *β*
  Bias operator
  Else (rand > *β*)
  Apply the transfer function operator
  End if
  End for

The article "Skin Cancer Detection Using Kernel Fuzzy C-Means and Improved Neural Network Optimization Algorithm" was published in 2021. Journal: Comput Intell Neurosci.

### 4.3. Improved Neural Network Algorithm

However, the neural network algorithm provides good results to solve different applications of optimization problems [20–22], and it is sometimes stuck in the premature convergence that gives a high impact on the solution accuracy. In this investigation, to modify this drawback, 2 mechanisms are considered. The first mechanism is to employ the Chaos theory. This mechanism explores novel situations, which are dynamic discrete-time, i.e.,

(14) $$\begin{array}{c} \beta_{m+1}=f\left(\beta_{m}\right),\;m=0,1,2,\ldots . \end{array}$$

In this research, the logistic map function has been used as the modification mechanism. This mechanism could be mathematically modeled as follows:

(15) $$\begin{array}{c} \beta_{j,i+1,q}=\rho \times \beta_{j,i,q}\left(1-\beta_{j,i,q}\right), \end{array}$$

where *i* signifies the populations' number, *β*_*j*,*i*,*q*_ defines the value for the *i*^th^ chaotic iteration, *ρ* describes a constant, which is set 4, *q* demonstrates the iteration number, *j* illustrates the generators' number in the system, and *β*_0_ describes the initial value of *β*_*i*_ with a random value between 0 and 1 [23, 24]. With assuming the above explanation, the set of initial variables *w*_*ij*_ is rewritten as follows:

(16) $$\begin{array}{c} w_{ij}=L_{j}+\left(U_{j}-L_{j}\right)\times \beta_{j,i,q}. \end{array}$$

This study also used Lévy flight (LF) as a second modification. The LF is a popular technique for improving optimization algorithms [25]. The LF uses random motion to control the local searching. This is obtained by the following equations:

(17) $$\begin{array}{c} Le\left(w\right)\approx \frac{1}{w^{1+\tau }},\\ w=\frac{A}{\sqrt[{\tau }]{\left|B\right|}},\\ \sigma^{2}={\left\{\frac{\Gamma \left(1+\tau \right)}{\tau \Gamma \left(\left(1+\tau \right)/2\right)}\times \frac{\sin\left(\pi \tau /2\right)}{2^{\left(1+\tau \right)/2}}\right\}}^{2/\tau }, \end{array}$$

where *τ* represents the Lévy flight index in the range [0, 2] (here, *τ*=1.5 [26]), *w* describes the step size, *A*, *B* ~ *N*(0, *σ*^2^), Γ(.) describes Gamma function, and the samples generate a Gaussian distribution with *σ*^2^ variance and zero mean value. By assuming the LF mechanism, the updated equation for the new pattern solutions based on the best weight value is achieved as follows:

(18) $$\begin{array}{c} W_{i}^{\text{updated}}\left(t+1\right)=W_{i}\left(t\right)+2\times \text{rand}\times \text{Le}\left(\delta \right)\times \left(W^{\text{Target}}\left(t\right)-W_{I}\left(t\right)\right). \end{array}$$

The article "Skin Cancer Detection Using Kernel Fuzzy C-Means and Improved Neural Network Optimization Algorithm" was published in 2021. Journal: Comput Intell Neurosci.

### 4.4. Algorithm Validation

To assess the effectiveness of the proposed improved neural network algorithm, six standard benchmark functions have been utilized, and the results are compared with some new state-of-the-art algorithms, containing multiverse optimizer (MVO) [27], moth-flame optimization (MFO) algorithm [28], world cup optimizer (WCO) [19], and the original neural network algorithm (NNA). The parameter settings of the algorithms are as follows: for MVO: wormhole existence probability (WEP); WEP_min_=0.2; WEP_max_=1; Coefficient(*P*)=6. For MFO: logarithmic spiral shaped(*b*)=1; for WCO: *α*=0.5, playoff=4%. The population size for whole algorithms is set to 100, and their maximum iteration is set to 100.  Table 1 tabulates the studied benchmark functions for the analysis. The benchmark functions are considered with 30 dimensions.

To validate the algorithms based on the studied functions, four statistical indicators including minimum amount (Min), maximum amount (Max), mean amount (Mean), and standard deviation amount (Std) are employed, and the results are indicated in Table 2.

According to Table 2, the outcomes of the suggested INNA have the proper outcomes in terms of lower, higher, and amount. Because it provides the minimum value for these values that is the main purpose of these benchmark functions, therefore, the proposed INNA has the highest accuracy. Furthermore, the proposed method with a minimum standard deviation value provides the highest reliable solution for the studied benchmark functions.

## 5. Feature Extraction and Selection Based on INNA

Feature selection is one of the most important methods and techniques for data preprocessing and data mining. Due to the introduction of new programs for large data mining, media information retrieval, and medical data processing that requires the processing of large volumes of data, it is important to limit the number of features. The purpose of feature extraction here is to take out the important characteristics from the region of interest in skin cancer images to simplify the diagnosis process. In this paper, 19 different features have been used for extraction from the image.  Table 3 indicates the used features for the extraction.

The article "Skin Cancer Detection Using Kernel Fuzzy C-Means and Improved Neural Network Optimization Algorithm" was published in 2021. Journal: Comput Intell Neurosci.

Therefore, here, we utilized a feature selection technique to reduce and select some more important features and to eliminate the low-cost features. Different methods have been introduced for this purpose. Metaheuristics are a kind of new technique for feature selection.

Feature selection using metaheuristics is one of the subsets of feature extraction and is discussed in various fields of machine learning and data mining. In general, this problem does not have a definite solution, and so far, no precise method has been proposed to solve it. Various classical approaches have been proposed to these problems, but usually, the quality of their solutions is generally not very good. In contrast, intelligent optimization methods can provide far better solutions to these problems. Therefore, one of the effective and constructive methods in solving feature selection problems and related issues is the use of metaheuristic optimization methods and evolutionary algorithms.

Here, we employed a cost function for optimum selection of the features using four indicators, including false positive (FP), false negative (FN), true positive (TP), and true negative (TN). The cost function is formulated as follows:

(19) $$\begin{array}{c} \text{fitness}=\frac{\left(\text{TP}\times \text{TN}\right)-\left(\text{FP}\times \text{FN}\right)}{\sqrt{\left(\left(\text{TN}+\text{FP}\right)\times \left(\text{TP}+\text{FP}\right)\times \left(\text{TP}+\text{FN}\right)\times \left(\text{TN}+\text{FN}\right)\right)}}. \end{array}$$

The idea is to minimize the abovementioned function with selecting the high cost and important features. Based on the designed INNA, the above function has been minimized, and less-cost features are eliminated from the processing. The next step is to employ an efficient method for classifying these features.

After performing the binary optimization technique on the features, the following features with higher effectiveness are selected for training: elongation, area, mean, correlation, entropy, and elongation. This selection is performed based on a metaheuristic technique based on a stochastic nature.

## 6. Skin Cancer Image Classification

Classification is the process of separating an input image into predetermined classes. Image classification is considered the last part of the diagnosis in medical image analysis. This step can decrease the time for the cancer diagnosis process by decreasing the search space in it. A popular and useful method in classification is to use a support vector machine (SVM). The SVM seeks the best hyperplane that operates as a multipart (here two-part) data separator in the input space. For reaching the constraints of the optimization problem, the support vector machine has been employed to evaluate the normal vector, *w*, in the hyperplane, the bias *b*, and the slack variable, *η* for incorrectly assigned training patterns that support the generalization, which is defined as follows:

(20) $$\begin{array}{c} y=\min\frac{w^{2}}{2}+C\times \sum_{i=1}^{n}\eta_{i}. \end{array}$$

With separation function:

(21) $$\begin{array}{c} y_{i}\left(q\times x_{i}+b\right)\geq 1-\eta_{i}. \end{array}$$

Feature space is highly affected by the separating function in equation (21), so that a function selection needs to be performed correctly to generate optimal output. Here, for minimizing equation (20), the suggested INNA has been utilized. Accordingly, the support vector machine uses a kernel that is employed to alter data to the feature space. In this research, three different kernels including linear, polynomial, radial basis function (RBF), and sigmoid have been used.  Figure 7 shows a typical SVM.

The article "Skin Cancer Detection Using Kernel Fuzzy C-Means and Improved Neural Network Optimization Algorithm" was published in 2021. Journal: Comput Intell Neurosci.

As can be explained, the SVM technique is a proper tool for classifying the images. Medical images are also a part of this event. Therefore, after performing feature extraction on the images for decreasing the operation complexity, the skin cancer features for each image can be injected into the SVM, and the SVM will present the final classification, which will be healthy or cancer.

## 7. Evaluation and Results

### 7.1. Implementation Details

As mentioned before, the proposed skin cancer detection system contains different modules that are generated in MATLAB R2019b environment. The modules include image segmentation, image acquisition, feature extraction and choice, and the last classification. In the image acquisition stage for dermoscopic images, American Cancer Society (ACS) [30] and PH^2^ [31] databases are used:

- The ACS database: the ACS database includes 68 pairs of XLM and TLM images that are integrated by the Nervoscope system. Experimental analysis is established by a 16 GB RAM Intel Core i7 processor. This database is downloaded one by one from https://www.cancer.org/cancer/skin-cancer.html.
- The PH^2^ database: dermoscopic images of this database are collected from the Dermatology Service of Hospital Pedro Hispano (Matosinhos, Portugal) under the same conditions. These images are 8-bit RGB color images with a resolution of 768 × 560 pixels. The image database includes a total of 200 dermoscopic images of melanocytic lesions, including 80 common nevi, 80 atypical nevi, and 40 melanomas. This database can be downloaded from: https://www.fc.up.pt/addi/ph2%20database.html.

The article "Skin Cancer Detection Using Kernel Fuzzy C-Means and Improved Neural Network Optimization Algorithm" was published in 2021. Journal: Comput Intell Neurosci.

The training and the test data for the benchmarks are set to 80% and 20%, respectively.

### 7.2. Results

As previously mentioned, the recommended simulations have been carried out to the ACS dataset to investigate the system efficiency. For numerical analysis of the suggested methodology, three popular measurement indicators for classification problems have been used. These metrics are accuracy (ACC), precision (PR), and sensitivity (SN). By comparing the ground-truth with the output mask, the classification indicators are evaluated as follows:

(22) $$\begin{array}{c} \text{ACC}=\frac{\text{TP}+\text{TN}}{\text{TP}+\text{TN}+\text{FP}+\text{FN}}\times 100,\\ \text{PR}=\frac{\text{TP}}{\text{TP}+\text{FP}}\times 100,\\ \text{SN}=\frac{\text{TP}}{\text{TP}+\text{FN}}\times 100, \end{array}$$

where TP, TN, FP, and FN denote the true positive, true negative, false positive, and false negative.

So, by analyzing the efficiency of the INNA-SVM method by considering different kernels based on the abovementioned indicators, we have the following.

It can be observed from Table 4 that the linear kernel of the proposed INNA-SVM, in addition to simplicity, results in the best values for all indicators for both databases: sensitivity, accuracy, and precision. Therefore, this kernel is utilized here for the classification of the features. For a comprehensive investigation about the proposed method's efficiency, five evaluation measurements including specificity (SP), positive predictive value (PPV), negative predictive value (NPV), F1 score, and Matthews correlation coefficient (MCC) are considered, which are mathematically as follows:

(23) $$\begin{array}{c} \text{SP}=\frac{\text{TN}}{\text{FP}+\text{TN}},\\ \text{PPV}=\frac{\text{TP}}{\text{TP}+\text{FP}},\\ \text{NPV}=\frac{\text{TN}}{\text{TN}+\text{FN}},\\ F1\text{ score}=\frac{2\times \text{TP}}{2\times \text{TP}+\text{FP}+\text{FN}},\\ MCC=\frac{\text{TP}\times \text{TN}-\text{FP}\times \text{FN}}{\sqrt{\left(\text{TP}+\text{FP}\right)\left(\text{TP}+\text{FN}\right)\left(\text{TN}+\text{FP}\right)\left(\text{TN}+\text{FN}\right)}}. \end{array}$$

The general proposed method has been compared with five new methods, and the comparison results have been indicated in Table 5. The compared methods include Astorino's method [5] based on multiple instance learning (MIL), Hassan's method [6] based on a simple pipeline image preprocessing technique, Barros's method [7] based on hardware designing by the multilayer perceptron, Santos's method [8] based on neural networks and fuzzy logic, and Wang's method [9] based on deep convolution networks. The results are achieved from the mean value of both databases.

The article "Skin Cancer Detection Using Kernel Fuzzy C-Means and Improved Neural Network Optimization Algorithm" was published in 2021. Journal: Comput Intell Neurosci.

According to Table 5, the F1-score of the suggested method with 84.39% that defines its accuracy based on the precision and recall of the test data is the highest among all of the compared methods. Also, the value of MCC in the proposed method with 94.21% is the highest among the others, and because it uses all of the analysis terms, it shows the method's higher efficiency than the others. Also, the higher value of the NPV and PPV with 95.57% and 85.09% against the other methods shows higher condition occurrence of the method to control the likelihood of a test identifying cancer toward the others. Finally, the higher SP value based on the proposed method reports higher occurrence-independent results of the algorithm.

## 8. Conclusions

Skin cancer is one of the most common cancers, and malignant melanoma is the most invasive and deadliest kind of this cancer. Early detection of this cancer by physicians has a high effect on the treatment of this cancer. Recently, several machine vision-based techniques are used for helping physicians with accurate early detection. This paper proposed a new approach for optimal skin cancer detection. The first section in the proposed method was to establish a preprocessing technique including noise reduction and contrast enhancement. Then, the region of interest (ROI) was segmented by a kernel fuzzy C-means segmentation method. The features of the ROI were then extracted, and the most important features were selected optimally. Afterward, the selected features were injected into an optimal classifier using support vector machine (SVM) for classification. The main contribution of this study was to present a developed version of a new metaheuristic, called neural network optimization algorithm, to optimize both parts of feature selection and SVM classifier in the system. The superiority of the proposed method was proved by performing a comparison among the suggested approach and five state-of-the-art methods.

## Figures and Tables

**Figure 1:** The statistical information of the lead cancers in (a) quantity and (b) death value in 2019 [4].

**Figure 2:** The flowchart of the suggested approach.

**Figure 3:** Image noise reduction: (a) image plus 0.1 salt and pepper noises and (b) image after noise reduction with median filtering.

**Figure 4:** (a) Original Image with low contrast. (b) Histogram of (A). (c) Contrast improvement of (A). (d) Histogram of (C).

The article "Skin Cancer Detection Using Kernel Fuzzy C-Means and Improved Neural Network Optimization Algorithm" was published in 2021. Journal: Comput Intell Neurosci.

**Figure 5:** Two sample examples of skin cancer segmentation based on the proposed KFCM methodology.

**Figure 6:** The structure of NNA.

**Figure 7:** A typical model of an SVM.

**Table 1:** The applied test functions for the analysis.

Function	Formula	Minimum	Limitation
Rosenbrock	*f*_1_=∑_*i*=1_^*D*−1^{100(*x*_*i*+1_ − *x*_*i*_)^2^+(*x*_*i*_ − 1)^2^}	0	[−30,30]^*D*^
Sum squares	*f*_2_=∑_*i*=1_^*D*^*ix*_*i*_^2^	0	[−10,10]^*D*^
Step 2	*f*_3_=∑_*i*=1_^*D*^(*x*_*i*_+0.5)^2^	0	[−100,100]^*D*^
Schwefel 2.22	*f*_4_=∑_*i*=1_^*D*^|*x*_*i*_| − ∏_*i*=1_^*D*^|*x*_*i*_|	0	[−10,10]^*D*^
Schwefel 1.2	*f*_5_=∑_*i*=1_^*D*^(∑_*j*=1_^*i*^*x*_*j*_)^2^	0	[−100,100]^*D*^
Chung Reynolds	*f*_6_=(∑_*i*=1_^*D*^*x*_*i*_^2^)^2^	0	[−100,100]^*D*^

**Table 2:** The simulation results of the comparative algorithms on the studied benchmark functions, moth-flame optimization (MFO) algorithm [28], world cup optimizer (WCO) [19], and the original neural network algorithm (NNA).

Algorithm		*f*_1_	*f*_2_	*f*_3_	*f*_4_	*f*_5_	*f*_6_
MVO [27]	Min	17.58	0.0024	0.0031	19.38	0	6.37*e* − 8
	Max	7.29*e* + 3	436.15	3.86*e* + 5	2.37*e* + 3	5.39*e* − 7	4.19*e* − 8
	Mean	2.96*e* + 3	280.16	4.19*e* + 4	67.25	6.15*e* − 9	1.27*e* − 7
	Std	5.79*e* + 2	95.37	6.37*e* + 4	11.62	3.19*e* − 8	3.07*e* − 7
MFO [28]	Min	28.14	2.57	0.051	6.29	4.38*e* − 6	8.39
	Max	129.08	4.18	9.27	53.49	0.015	110.35
	Mean	80.46	23.09	4.52	30.17	0.02	35.08
	Std	22.46	1.64	1.73	3.28	0.01	24.63
WCO [19]	Min	7.39	5.13*e* − 5	5.92*e* − 5	2.57	1.94*e* − 8	6.38*e* − 9
	Max	1.38*e* + 2	0.264	0.017	4.12	7.51*e* − 8	7.29*e* − 8
	Mean	105.37	0.0573	0.024	3.28	6.48*e* − 9	1.18*e* − 9
	Std	14.83	0.0873	3.28*e* − 5	1.23	4.29*e* − 9	3.19*e* − 8
NNA [29]	Min	4.91	6.29*e* − 21	9.75*e* − 9	0.017	9.37*e* − 16	5.9*e* − 17
	Max	45.22	34.39*e* − 18	1.19*e* − 8	4.62	2.58*e* − 12	5.19 *e* − 16
	Mean	13.83	6.30*e* − 18	5.94*e* − 8	0.532	3.42*e* − 13	6.67*e* − 16
	Std	5.29	3.62*e* − 21	6.53*e* − 9	0.42	1.97*e* − 13	7.50*e* − 17
INNA	Min	5.16	15.26*e* − 22	6.37*e* − 11	6.38*e* − 15	7.26*e* − 7	6.71*e* − 39
	Max	111.57	6.76*e* − 20	4.29*e* − 10	3.95*e* − 14	0.0234	9.43*e* − 35
	Mean	24.13	2.48*e* − 20	1.17*e* − 10	1.09*e* − 14	3.11*e* − 5	4.57*e* − 6
	Std	12.28	6.19*e* − 21	5.64*e* − 11	9.64*e* − 15	11.97*e* − 7	9.55*e* − 36

**Table 3:** Utilized features for the extraction.

Parameter	Equation	Parameter	Equation
Elongation	$\sqrt{\text{number of tumor pixels}/2\times {\left(\text{Max radius}\right)}^{2}}$	Compactness	$\left(2\times \sqrt{\text{number of tumor pixels}\times \pi }\right)/\text{Area}$
Area	∑_*i*=1_^*M*^∑_*j*=1_^*N*^*p*(*i*, *j*)	Mean	1/MN(∑_*i*=1_^*M*^∑_*j*=1_^*N*^*p*(*i*, *j*))
Perimeter	∑_*I*=1_^*M*^∑_*j*=1_^*N*^*B*_*p*_(*i*, *j*)	Correlation	∑_*i*=1_^*M*^∑_*j*=1_^*N*^*p*(*i*, *j*) − *μ*_*r*_*μ*_*c*_/*σ*_*r*_*σ*_*c*_
Variance	1/MN(∑_*i*=1_^*M*^∑_*j*=1_^*N*^(*p*(*i*, *j*) − *μ*))	Solidity	Area/convex area
Invariant moments	*φ*_1_=*η*_20_+*η*_02_	Entropy	−∑_*i*=1_^*M*^∑_*j*=1_^*N*^*p*(*i*, *j*)log*p*(*i*, *j*)
	*φ*_2_=(*η*_20_ − *η*_02_)^2^+4*η*_11_^2^		
	*φ*_3_=(*η*_30_ − 3*η*_12_)^2^+(3*η*_21_ − *μ*_03_)^2^		
Elongation	$2\sqrt{\text{Area}}/a\sqrt{\pi }$	Eccentricity	2*a*^−1^(*a*^2^ − *b*^2^)^0.5^
Rectangularity	Area/*b* × *a*	Energy	∑_*i*=1_^*M*^∑_*j*=1_^*N*^*p*^2^(*i*, *j*)
Irregularity index	4*π* × area/perimeter^2^	Standard deviation	Variance^1/2^
Form factor	Area/a^2^		

MN describes the image size, *B*_*p*_ defines the external side length for the boundary pixel, *p*(*i*, *j*) defines the pixels intensity amount at position (*i*, *j*), *μ* and *σ* describe the mean value and the standard deviation, orderly, and *a* and *b* present the major axis and the minor axis, respectively. However, some of the above features have a high impact, and some others have a low impact on feature extraction.

The article "Skin Cancer Detection Using Kernel Fuzzy C-Means and Improved Neural Network Optimization Algorithm" was published in 2021. Journal: Comput Intell Neurosci.

**Table 4:** The classification results of INNA-SVM method based on different kernels in two databases.

Database	Kernel	ACC (%)	Pr (%)	SN (%)
ACS [30]	Linear	64.19	65.18	64.19
	RBF	37.57	38.09	37.57
	Polynomial	46.29	38.61	46.29
	Sigmoid	40.16	41.53	40.16
PH^2^ [31]	Linear	70.00	69.00	71.00
	RBF	42.00	43.00	42.00
	Polynomial	51.00	45.00	51.00
	Sigmoid	42.50	46.00	53.00

**Table 5:** The performance comparison between the suggested method and the analyzed methods.

Method	MCC (%)	SP (%)	PPV (%)	NPV (%)	*F*1-score (%)
The proposed method	92.35	88.67	81.43	92.66	81.69
Astorino's method [5]	72.29	87.49	81.37	86.72	69.29
Hassan's method [6]	75.46	80.76	69.35	85.87	63.49
Barros's method [7]	83.65	60.34	68.37	83.98	70.81
Santos's method [8]	85.74	60.41	71.95	86.69	76.76
Wang's method [9]	88.67	80.77	74.49	83.71	82.92

## Data Availability

The data are available at https://www.cancer.org/.
